The article "Single-Cell Transcriptome Analysis Reveals the Importance of IRF1/FSTL1 in Synovial Fibroblast Subsets for the Development of Rheumatoid Arthritis" was retracted in 2023. Reasons: signs of a paper mill; compromised peer review; unreliable results or conclusions.

# Single-Cell Transcriptome Analysis Reveals the Importance of IRF1/FSTL1 in Synovial Fibroblast Subsets for the Development of Rheumatoid Arthritis

**DOI:** 10.1155/2022/1169614

**Published:** 2022-05-05

**Authors:** Qiang Wang, Xia Yu, Mingzhi Gong

**Affiliations:** ^1^Department of traumatic orthopedics, The Second Hospital, Cheeloo College of Medicine, Shandong University, Jinan, Shandong 250012, China; ^2^Department of Joint and Sports Medicine, Taian City Central Hospital, Taian City, Shandong, China; ^3^Department of nuclear medicine, Taian City Central Hospital, Taian City, Shandong, China

## Abstract

**Objectives:**

This study aimed to investigate the potential role of synovial fibroblasts (SFs) in the development of rheumatoid arthritis (RA) to identify potential molecular targets and provide a theoretical basis for the treatment of RA.

**Methods:**

GSE109449, a fibroblast transcriptome dataset of synovial tissue from RA and osteoarthritis (OA), were obtained from the GEO database. After standard cell quality control, this single-cell transcriptome data was used to perform routine single-cell analysis processes. After completing dimensionality reduction, clustering, and cell subset identification of fibroblasts, the SCENIC analysis helped calculate the significant gene regulatory networks in fibroblasts and their subsets. From these computed gene regulatory networks, the regulon in which follistatin-like protein 1 (FSTL1) resides was extracted and used to analyze the transcriptional regulatory status of fibroblasts. Finally, the gene set enrichment analysis (GSEA) was used to calculate the respective enriched gene sets of IRF1 and FSTL1.

**Results:**

Three SF subgroups were identified from the single-cell transcriptome analysis; SF subset 3 was more abundant in RA than in OA (*p* < 0.001). From the SCENIC analysis, we obtained 269 regulons and the corresponding gene regulatory networks in SF from the RA datasets. Next, we screened and obtained a regulon-containing FSTL1, where IRF1 was the major transcription factor. The top five regulons in SF subset 3 were TWIST1, MECOM, KLF6, MAFB, and RUNX1. Among the 3 SF subsets, IRF1 regulon was ranked the highest in SF subset 3. Differential analysis of pseudobulk RNA-seq showed that IRF1 was up-regulated in RA compared to OA. Between the three SF subgroups, IRF1 and FSTL1 expression was more up-regulated in SF subset 3 compared to the other two subgroups.

**Conclusions:**

IRF1 was found to regulate the invasiveness of SFs by regulating FSTL1, which may influence the disease progression of RA.

## 1. Background

Rheumatoid arthritis (RA) is a chronic immune disease characterized by synovial involvement and bone destruction, and its pathology is dominated by chronic synovitis [1]. The prevalence of RA is gradually expanding due to increased life expectancy and the high incidence of RA in older age groups [2]. The clinical symptoms in patients with RA are similar to those of inflammatory arthritis [3]. The prominent ones being are morning stiffness and pain, and in severe cases, joint dysfunction, resulting in a severe deterioration in their quality of life. Currently, a lot of mechanism is still unknown about the development of RA. However, a combination of genetic and environmental factors may contribute to the progression of RA.

The article "Single-Cell Transcriptome Analysis Reveals the Importance of IRF1/FSTL1 in Synovial Fibroblast Subsets for the Development of Rheumatoid Arthritis" was retracted in 2023. Reasons: signs of a paper mill; compromised peer review; unreliable results or conclusions.

At the cellular level, the typical pathology of RA is a persistent proliferation of synovial fibroblast (SF) in the joints and the formation of sarcomeres. SF is the most common cell type in the articular cartilage junction and is produced by bone marrow mesenchymal cells. In RA, SF is characterized by excessive proliferation, reduced apoptosis, increased cell migration, and invasiveness. It is highly invasive to the extracellular matrix and exacerbates joint damage [4]. Further, it can cause chronic synovitis in joints by producing and releasing inflammatory cytokines, chemokines, and matrix-degrading molecules. Subsequently, it can migrate to and invade the articular cartilage, thereby eroding and destroying it [5, 6]. SF can be a potential and safe therapeutic target for the treatment of RA [7]. Therefore, understanding the principal factors and their gene regulatory networks in SF involved in the development of RA is essential for designing novel and effective therapeutic strategies.

Follistatin-like protein 1 (FSTL1) is an extracellular matrix glycoprotein that promotes endothelial cell and vascular regeneration in response to ischemic stress and is thought to be an inflammatory indicator. Elevated levels of FSTL1 have been found in mouse models of collagen-induced arthritis [8]. In addition, high FSTL1 levels are associated with the poor prognosis of RA and also reflect systemic levels of inflammation in autoimmune diseases [9]. During the development of RA, FSTL1 overexpression promotes cell proliferation, migration, and invasiveness of the extracellular matrix of SF through increased expression of TLR4 and NF*κ*B [10, 11]. Antagonism against FSTL1 exerts an effective antifibrotic effect and reduces the severity of arthritis [12]. Therefore, elucidating the transcription factors (TFs) and gene regulatory networks regulating FSTL1 will likely lead to the development of novel therapeutic approaches for RA. In recent years, the advent of single-cell RNA sequencing (scRNA-seq) technology has enabled us to access the overall transcriptome expression data of a single cell to study the molecular interactions and regulation at the single-cell level. In comparison to bulk RNA, scRNA-seq analysis enables high-throughput analysis of cellular transcriptome expression at the single-cell level, opening a new window into the study of multicellular biological heterogeneity. In RA, scRNA-seq has allowed researchers to identify synovial cell types and study cell differentiation and development around cell subpopulations to explore novel therapeutic targets [13].

The article "Single-Cell Transcriptome Analysis Reveals the Importance of IRF1/FSTL1 in Synovial Fibroblast Subsets for the Development of Rheumatoid Arthritis" was retracted in 2023. Reasons: signs of a paper mill; compromised peer review; unreliable results or conclusions.

In this study, we aimed to investigate the potential role of SF in the development of RA and the important regulons associated with FSTL1 in it. We believe that this study will help us search for potential therapeutic targets and provide a theoretical basis for the therapeutic targets in RA, which can ultimately improve the quality of life of RA patients.

## 2. Methods

### 2.1. Data Acquisition and Preprocessing

We applied the keyword “rheumatoid arthritis” to search the GEO database. Then, we filtered the retrieved results to obtain a dataset containing scRNA-seq data of RA samples. Based on our pre-established criteria, a GSE109449 [14] dataset containing transcript data of 384 fibroblasts from four synovial tissues met our screening criteria and was included in the study. We then applied the “Seurat” package [15] for quality control of this scRNA-seq data. Cell damage or library preparation failure (invalid reverse transcription or PCR amplification failure) often introduces some low-quality data during cell isolation. The main features of the low-quality data are (i) low counts on the cells as a whole; (ii) low expression of genes; and (iii) a relatively high proportion of mitochondrial genes. If low-quality cells are not removed, it may affect downstream analysis (e.g., normalization, differential expression, and cell classification). So, we make sure to remove these low-quality cells and genes before performing the analysis. Therefore, those cells with gene expression type >1000, mitochondrial gene expression <15%, and hemoglobin-related genes <1% were screened for subsequent analysis. Our parameter settings refer to the recommendations of the previous studies [16–19].

### 2.2. Single-Cell Analysis and Identification of Fibroblast Subpopulations

After the single-cell transcriptome data in count format were normalized, the “FindVariableFeatures” function was used to find the 2000 highly variable genes in the header. Subsequently, by applying the “RunPCA” function, we linearly transformed the single-cell transcriptome data to extract the principal components (PCs). Considering the heterogeneity among different batches of samples, we applied the “harmony” R package to de-batch the data. Among them, we selected the top 15 PCs for downscaling and clustering and applied the uniform manifold approximation and projection (UMAP) [20] to visualize the cell clustering results. We projected the subgroups of SFs identified in the original study onto our UMAP and further identified three SF subgroups from them. We then applied the SCENIC tool to analyze the key transcriptional regulatory networks in these three SF subgroups.

The article "Single-Cell Transcriptome Analysis Reveals the Importance of IRF1/FSTL1 in Synovial Fibroblast Subsets for the Development of Rheumatoid Arthritis" was retracted in 2023. Reasons: signs of a paper mill; compromised peer review; unreliable results or conclusions.

### 2.3. SCENIC and Gene Regulatory Networks

SCENIC is a computational tool that allows gene regulatory network identification from single-cell transcripts based on cellular states [21]. To further explore the functional differences of the three SF subsets, we applied pySCENIC v. 0.11 (a python implementation of the SCENIC pipeline) to mine the TFs and their corresponding gene regulatory networks in SFs. First, single-cell transcriptome data were used to construct a gene coexpression network. Subsequently, RcisTarget was used to identify TFs and the genes they directly regulate. The regulatory interactions between regulators and their potential targets constitute a gene regulatory network. From the gene regulatory network, we can mine the key TFs that regulate the genes of interest [22]. Based on the gene regulatory network, the regulon activity score (RAS) was calculated to quantify the regulatory capacity of regulons in the cell. Subsequently, a regulon specificity score (RSS) was further calculated to characterize the regulatory activity of regulons in cell subtypes, and all regulons in each cell subtype were ranked from the largest to the smallest according to the size of RSS. The genes in the regulatory network regulated by key TFs were further predicted in STRING (https://cn.string-db.org/), and the protein-protein interaction (PPI) network was constructed.

### 2.4. Differential Expression Analysis

Differential gene expression analysis was performed in SFs between the RA and OA groups. Using the single-cell transcriptome data, we detected the differentially expressed genes (DEGs) in all SFs by the “FindMarker” function. Further, to explore the relevant DEGs at the bulk RNA level, we performed pseudobulk RNA analysis [23]. First, the RNA count values of each gene were summed for all cells in each sample to estimate the corresponding gene expression at the bulk RNA-seq level. Then, DESeq2 [24] was used to perform differential expression analysis on the constructed pseudobulk transcript data.

### 2.5. Functional Pathway Analysis

Functional pathway analysis included the Kyoto Encyclopedia of Genes and Genomes (KEGG) and gene ontology (GO), which were analyzed by the clusterProfiler R package [25, 26]. Gene set enrichment analysis (GSEA) was used to explore the functional pathways enriched by the dysregulated molecules. We selected c2.cp.v7.2.symbols.gmt [Curated] as the reference gene set for GSEA [27].

The article "Single-Cell Transcriptome Analysis Reveals the Importance of IRF1/FSTL1 in Synovial Fibroblast Subsets for the Development of Rheumatoid Arthritis" was retracted in 2023. Reasons: signs of a paper mill; compromised peer review; unreliable results or conclusions.

### 2.6. Statistical Methods

Most analyses and graphical plots were performed using R (v. 4.0.2). All tests were two-sided, and *p* < 0.05 was considered statistically significant. Two single-cell clustering approaches, UMAP and tSNE, were used concurrently in this investigation. This is because they each have their own distinct advantages: (i) UMAP employs an exponential probability distribution in high dimensions, whereas tSNE is limited to Euclidean distance; (ii) UMAP employs binary cross-entropy (CE) as the cost function, rather than K-L scatter as in tSNE; and (iii) UMAP employs the graph Laplace transform to initialize low-dimensional coordinates, as opposed to tSNE's random normal initialization.

Thus, for the transcriptional regulatory network analysis, we employed the tSNE clustering approach, whereas for the cell type clustering analysis, we used the UMAP method. Both UMAP and tSNE clustering analyses performed well in this investigation, which further demonstrates the beneficial effect of hierarchical clustering in this study.

## 3. Results

### 3.1. Quality Control of Single-Cell Transcripts

Based on the characteristic distribution of the single-cell data in this dataset (Figure 1(a)), we set filtering conditions to control the cell quality. The data quality of the filtered cells is shown in Figures 1(b)–1(f). A total of 371 cells met the filtering criteria and were used for subsequent analysis. We further identified the top 2000 highly variable genes from those genes that were expressed in at least three cells. Subsequently, based on these highly variable genes, the single-cell data were downscaled and presented in UMAP (Figures 1(a) and 1(b)).  Figure 1(g) shows the single-cell data of the four samples after downscaling. The clustering results showed that the four samples were well integrated, indicating that batch effects between samples were removed.  Figure 1(h) shows the proportion of cell distribution between OA and RA groups.

### 3.2. Identification of Three Synovial Fibroblast Subsets

The relationship between the clustering results of single-cell data and the chosen resolution is shown in Figure 2(a). As the resolution was set from 0.01 to 1, the corresponding number of cell clusters varied from 2 to 7. We chose a resolution of 0.5 for the final clustering and obtained four cell clusters (Figure 2(b)). The distribution of cellular features in these four clusters is shown in Figures 2(c) and 2(d). The variability in the number of genes and mitochondrial gene expression was higher in cluster 2 than in the other three clusters. The distribution of cellular features in clusters 1 and 3 was more consistent. Subsequently, we projected the three fibroblast subpopulations (CD34-THY-, CD34-THY+, and CD34+) identified in the original study onto UMAP (Figure 2(e)) [14]. Between the OA and RA groups, the cell population presented three types of cell subpopulations. Combined with the dynamic clustering tree (Figure 2(a)), we named cluster 0 as SF subset 1 (SF_1), cluster 2 as SF subset 2 (SF_2), and clusters 1 and 3 as SF subset 3 (SF_3) (Figure 2(f)). The proportions of these three SF subsets in the four samples are shown in Figure 2(g). The proportion of SF subset 1 in RA was lower relative to that in OA (17.9% versus 55.6% in RA and OA, respectively, *p* < 0.001). Further, the proportion of SF subset 3 in RA was elevated relative to that in OA (56.5% versus 16.6% in RA and OA, respectively, *p* < 0.001). Although in SF subset 3, the expression of IRF1 and FSTL1 did not differ significantly between the RA and OA groups, the proportion of SF subset 3 was significantly higher in the RA than in the OA group. This suggested that SF subset 3 may be a critical SF subgroup involved in the development of RA.

The article "Single-Cell Transcriptome Analysis Reveals the Importance of IRF1/FSTL1 in Synovial Fibroblast Subsets for the Development of Rheumatoid Arthritis" was retracted in 2023. Reasons: signs of a paper mill; compromised peer review; unreliable results or conclusions.

### 3.3. IRF1–FSTL1 Identified by SCENIC

From the given single-cell transcriptome data and cell states, SCENIC identified 269 regulons in the three SF subsets. Subsequently, RcisTarget was used to identify TFs and the genes they directly regulate. The regulatory interactions between regulators and their potential targets constitute a gene regulatory network. Of these, FSTL1 was found in the interferon regulatory factor 1 (IRF1-)-regulated gene regulatory network. We used t-distributed stochastic neighbor embedding (t-SNE) [28] to show the results of cell clustering in the SCENIC analysis process. The distribution of the three SF subsets in tSNE is shown in Figures 3(a)–3(c), while the distribution of cell clusters in tSNE is shown in Figure 3(d). Based on RSS, the regulons in each cell subpopulation were arranged from large to small. The top five regulons in each SF subset and the IRF1 sorting position were different among the three SF subsets (Figures 3(e)–3(g)). In SF subset 1, the top five regulons were CUX1, MAFK, DLK4, SIX3, and KLF12. In SF subset 2, the top five regulons were HNF1B, ZNF71, ELF5, PAX4, and TAL1, while in SF subset 3, the top five regulons were TWIST1, MECOM, KLF6, MAFB, and RUNX1. Thus, there is heterogeneity in transcriptional regulation among the three identified SF subgroups. Among the three subgroups, IRF1 had the highest alignment in SF subset 3, indicating that IRF1 has different regulatory activities among the SF subgroups. For the gene regulatory network regulated by IRF1, the constructed core PPI network is illustrated in Figure 3(h), which shows the important molecules related to IRF1.

The article "Single-Cell Transcriptome Analysis Reveals the Importance of IRF1/FSTL1 in Synovial Fibroblast Subsets for the Development of Rheumatoid Arthritis" was retracted in 2023. Reasons: signs of a paper mill; compromised peer review; unreliable results or conclusions.

### 3.4. Pseudobulk RNA-seq Analysis Showed That IRF1 Was Up-regulated in RA

Based on SF pseudobulk transcripts, differential analysis between the OA and RA groups showed that IRF1 was up-regulated in RA (Figure 4(a)). Among them, 1100 up-regulated and 1398 down-regulated genes were identified in RA and were included in GO and KEGG functional pathway analyses. The up-regulated genes in RA compared to OA were enriched in mesenchymal cell development, mesenchymal cell differentiation, and stem cell development (Figure 4(b)). Further, immune and ossification functions were up-regulated in OA. In contrast, graft-versus-host disease, the intestinal immune network for IgA production, extracellular matrix structural constituent, and ossification pathways were down-regulated in RA (Figure 4(c)). Differential analysis at the single-cell level also showed that IRF1 was up-regulated in RA (Figure 4(d)). The top 20 up-regulated and down-regulated DEGs in SFs between RA and OA are shown in a heat map (Figure 4(e)).

### 3.5. Key Regulons in the Synovial Fibroblast Subsets

To explore the differences in gene regulatory networks in the SF subset between RA and OA groups, we analyzed the key regulons in the three SF subsets. The distribution of SF subset 1 in tSNE is shown in Figure 5(a). The top five regulons in SF subset 1 and the IRF1 sorting positions were different between RA and OA (Figures 5(b)–5(c)). The top five regulons in the RA group were MAFK, CUX1, PAX8, RB1, and SNAPC5, while the top five regulons in the OA group were CUX1, MAFK, DLX4, HES1, and SIX3. The RSS ranking of IRF1 in the RA group was higher than that in the OA group. According to SCENIC analysis, SFs regulated by IRF1 were shown in tSNE (Figure 5(d)). In addition, differential analysis at the single-cell sample level showed that IRF1 was up-regulated and FSTL1 was down-regulated in the RA group compared to the OA group (Figure 5(e)).

The same analysis was also applied to SF subsets 2 and 3 (Figures 5(f)–5(i) and Figures 6(a)–6(c)). Similarly, we found that in both SF subsets 2 and 3, the ranking of IRF1 was higher in RA than in the OA group. Differential expression analysis showed that in SF subset 2, IRF1 was not different between the two groups, while FSTL1 was down-regulated in the RA group (Figure 5(f)). In SF subset 3, both IRF1 and FSTL1 were not significantly different between the OA and RA groups (Figure 6(d)). The expression of IRF1 and FSTL1 in the three SF subsets is shown in UMAP (Figure 6(e)). From this, we found that in RA, IRF1 and FSTL1 were significantly enriched mainly in SF subset 3. The above results showed the heterogeneity at the level of transcriptional regulation between the RA and OA groups in the three identified SF subsets.

The article "Single-Cell Transcriptome Analysis Reveals the Importance of IRF1/FSTL1 in Synovial Fibroblast Subsets for the Development of Rheumatoid Arthritis" was retracted in 2023. Reasons: signs of a paper mill; compromised peer review; unreliable results or conclusions.

### 3.6. Possible Functions of IRF1 and FSTL1

GSEA was used to explore the possible functions of IRF1 and FSTL1. In the samples with elevated IRF1, oxidation by cytochrome P450, citrate cycle (tri-carboxylic acid cycle), glucocorticoid biosynthesis, and neuroactive ligand-receptor interaction were up-regulated, while the metabolism of angiotensinogen to angiotensin was down-regulated (Figure 6(f)). In the samples with up-regulated FSTL1, mitochondrial tRNA aminoacylation, type I collagen synthesis in the context of osteogenesis imperfecta, and oxidative phosphorylation were up-regulated, while neuroactive ligand-receptor interaction was down-regulated (Figure 6(g)). Thus, IRF1 may be involved in steroid hormone synthesis, while FSTL1 may be crucial for collagen synthesis and enhanced oxidative phosphorylation in RA.

## 4. Discussion

In this study, we explored the role of SF in the progression of RA. Three SF subsets were identified from RA synovial fibroblasts, and SF subset 3 was critical for promoting RA progression. IRF1 was found to regulate the invasiveness of SFs by regulating FSTL1, which may influence the disease progression of RA.

Combined with SCENIC analysis, we analyzed the regulons and corresponding gene regulation sets in the SFs, thus unraveling the transcriptional patterns of SFs in RA. FSTL1 was present in the regulon regulated by IRF1. Inflammatory cytokines can promote the nuclear localization of IRF1, which enhances the transcription of a subset of type I interferon response genes, thereby promoting RA progression [29]. Subsequently, we screened and obtained a regulon-containing FSTL1, in which IRF1 was identified as the major TF. Pseudobulk RNA analysis revealed that IRF1 expression was up-regulated in SFs in RA compared to that in OA. Furthermore, functional pathway analysis in RA and OA revealed that cell development and differentiation pathways were up-regulated in RA, including mesenchymal cell differentiation and development. Thus, SFs in RA exhibited a more proliferative cellular profile relative to SFs in OA. PPI network analysis of the IRF1 regulon showed significant interactions between IRF1 and STAT2, HLA-E, HLA-B, and HLA-F. Among them, STAT2 and STAT6 are thought to be associated with autoimmune diseases [30]. In addition, FSTL1 promotes the secretion of different matrix metalloproteases through the activation of MAPK, JAK/STAT3, and NF-*κ*B pathways, thus accelerating the progression of RA [8].

The article "Single-Cell Transcriptome Analysis Reveals the Importance of IRF1/FSTL1 in Synovial Fibroblast Subsets for the Development of Rheumatoid Arthritis" was retracted in 2023. Reasons: signs of a paper mill; compromised peer review; unreliable results or conclusions.

SF subset analysis showed significant intercellular heterogeneity. Compared to the OA group, the proportion of SF subset 1 was significantly decreased while that of SF subset 3 was increased in the RA group. In SF subset 1, IRF1 expression was higher in the RA group than in the OA group. Although in SF subset 3, the expression of IRF1 and FSTL1 did not differ significantly between the RA and OA groups, the proportion of SF subset 3 was significantly higher in the RA than in the OA group. This suggested that SF subset 3 may be a critical SF subgroup involved in the development of RA. The most prominent regulons in SF subset 3 were TWIST1, MECOM, KLF6, MAFB, and RUNX1. Among these three subgroups, the RSS of IRF1 regulon had the highest alignment with SF subset 3, indicating that IRF1 plays a critical transcriptional regulatory role in SF subset 3. In addition, among the three SF subsets, the expression of IRF1 and FSTL1 was more pronounced in SF subset 3 compared to the other two subsets. In summary, IRF1 may control the severity of RA in SF by regulating FSTL1. The high number of cells affected by IRF1 regulation in SF subset 3 could lead to an increased progression of RA. The analysis of SF subsets will allow us to target the right subset of cells to develop novel treatment strategies against RA. GSEA showed that oxidation by cytochrome P450, citrate cycle, and glucocorticoid biosynthesis pathways, which are associated with sterol hormone synthesis, were up-regulated in cells with elevated IRF1 expression. In cells with a high FSTL1 expression, pathways associated with enhanced collagen synthesis and oxidative phosphorylation were up-regulated. We speculate that the up-regulation of these pathways may provide the necessary conditions for the invasiveness of SF to the extracellular matrix.

Single-cell technology has been found to play a major role in the uncovering of regulatory networks in recent years. Rheumatoid arthritis (RA) is a chronic immune disease highly prevalent among the elderly. RA is characterized by a persistent proliferation of the synovial fibroblast (SF) cells. Hence, understanding the principal factors and their gene regulatory networks in SF involved in the development of RA is essential for designing novel and effective therapeutic strategies. Three SF subsets in RA were identified by applying single-cell transcriptome analysis in this research. We then analyzed the transcriptional regulatory network in the SF subsets and selected the regulon where FSTL1 was located for further analysis. SF subset 3 was identified as a pathogenic cell subset that promoted RA progression. By exploring this cell subset for therapeutic targets, we may find therapeutic modalities to improve the quality of life of RA patients. However, there are several limitations of our study. First, the lack of normal tissue samples in this acquired single-cell transcriptome dataset led us to obtain only differential genes between disease states, which would limit the results of the analysis. Next, the conclusions obtained from bioinformatics analysis in this study lack validation by biological experiments. We also combined single-cell analysis and gene regulation analysis to identify new cell subpopulations from SF and analyze their major transcriptional regulators and the genes they regulate. In the future, further experiments are needed to investigate the mechanism of the roles of IRF1 and FSTL1 on joint damage in the RA patient population.

The article "Single-Cell Transcriptome Analysis Reveals the Importance of IRF1/FSTL1 in Synovial Fibroblast Subsets for the Development of Rheumatoid Arthritis" was retracted in 2023. Reasons: signs of a paper mill; compromised peer review; unreliable results or conclusions.

## 5. Conclusion

We identified three SF subsets in RA and found that SF subset 3 may be critical for promoting RA progression. This SF subset 3 was more influenced by IRF1 regulation than the other two SF subsets. IRF1 regulated the aggressiveness of SFs by controlling FSTL1. This resulted in the modulation of the severity of RA. Notably, further experiments are needed to verify these bioinformatics findings.

## Figures and Tables

**Figure 1:** UMAP visualization showing the downscaling of scRNA-seq data from synovial fibroblasts. (a) Scatter plot showing single-cell quality control before data filtering. (b–f) Quality control of single-cell transcriptome data after data filtering. (g) UMAP shows the distribution of single cells between samples after downscaling. (h) UMAP shows the distribution of single cells between OA and RA groups.

**Figure 2:** Clustering of single-cell transcriptome data. (a) Dynamic clustering tree showing the process of clustering of cell clusters as the resolution changes. (b) UMAP illustrates the comparison of the distribution of cell clusters between OA and RO. (c–d) Quality control of single-cell transcriptome data in four cell clusters after clustering. (e) UMAP shows the comparison between OA and RA groups for SF subgroups from the original study. (f) UMAP displays the distribution of the three SF subsets between the two groups. (g) Bar chart showing the percentage of three SF subsets in each of the four samples.

**Figure 3:** SCENIC analysis showing the presence of FSTL1 in the IRF1 regulon in SFs. (a–c) tSNE shows the distribution of the three SF subsets in the SCENIC analysis. (d) tSNE shows the distribution of the four cell clusters in SCENIC obtained in the single-cell analysis. (e–g) The top five regulons of the three SF subsets and the sorted position of the IRF1 regulon. (h) PPI network calculated from STRING shows the molecules associated with IRF1.

The article "Single-Cell Transcriptome Analysis Reveals the Importance of IRF1/FSTL1 in Synovial Fibroblast Subsets for the Development of Rheumatoid Arthritis" was retracted in 2023. Reasons: signs of a paper mill; compromised peer review; unreliable results or conclusions.

**Figure 4:** Variance analysis and functional pathway analysis. (a) Volcano plot showing differentially expressed genes between RA and OA groups. Among them, IRF1 expression is up-regulated in RA relative to that in OA. (b–c) Pathway enrichment analysis showing (b) up-regulated and (c) down-regulated pathways in RA. (d) Analysis of gene expression differences between RA and OA groups at the single-cell level. Yellow dots represent genes up-regulated in RA, and dark blue dots represent genes up-regulated in OA. Large diameter dots represent genes that are differentially expressed between the two groups. (e) Heat map showing the expression of top 20 up-regulated and top 20 down-regulated genes of the RA and OA groups.

**Figure 5:** Comparison of regulon between the RA and OA groups. (a) In the SCENIC analysis, tSNE of the distribution of SF subset 1 between the RA and OA groups. (b–c) The top 5 regulons and IRF1 regulon of both RA and OA groups are ranked based on the RSS ranking position. (d) Regulatory status of the IRF1 regulon in single cells. (e–f) Analysis of gene expression differences between RA and OA groups at the single-cell level. Yellow dots represent genes up-regulated in RA and dark blue dots represent genes up-regulated in OA. Large diameter dots represent genes that are differentially expressed between the two groups. (g) The tSNE of the distribution of SF subset 2 between the RA and OA groups. (h–i) The top 5 regulons and IRF1 regulon of both RA and OA groups were ranked based on the RSS ranking position.

**Figure 6:** Expression of IRF1 and FSTL1 between OA and RA groups and GSEA. (a) In the SCENIC analysis, tSNE of the distribution of SF subset 1 between the RA and OA groups. (b–c) The top 5 regulons and IRF1 regulon of the RA and OA groups were ranked based on RSS. (d) Analysis of gene expression differences between RA and OA groups at the single-cell level. (e) Expression of IRF1 and FSTL1 between OA and RA groups. (f–g) GSEA of ARF1 and FSTL1.

## Data Availability

The data for this study were obtained from the GSE109449 dataset of the GEO database.

## Abbreviations

(RA): Rheumatoid arthritis
(scRNA-seq): Single-cell RNA sequencing
(SF): Synovial fibroblast
(FSTL1): Follistatin-like protein 1
(TFs): Transcription factors
(IRF1): Interferon regulatory factor 1
(UMAP): Uniform manifold approximation and projection
(t-SNE)L: T-distributed stochastic neighbor embedding
(SCENIC): Single-cell regulatory network inference and clustering.
